The article "Downregulation of uPAR and Cathepsin B Induces Apoptosis via Regulation of Bcl-2 and Bax and Inhibition of the PI3K/Akt Pathway in Gliomas" was retracted in 2020. Reasons: fabricated or falsified data; an official misconduct investigation; misconduct by an author; duplicated images.

# Downregulation of uPAR and Cathepsin B Induces Apoptosis via Regulation of Bcl-2 and Bax and Inhibition of the PI3K/Akt Pathway in Gliomas

**DOI:** 10.1371/journal.pone.0013731

**Published:** 2010-10-29

**Authors:** Ramarao Malla, Sreelatha Gopinath, Kiranmai Alapati, Christopher S. Gondi, Meena Gujrati, Dzung H. Dinh, Sanjeeva Mohanam, Jasti S. Rao

**Affiliations:** 1 Department of Cancer Biology and Pharmacology, University of Illinois College of Medicine at Peoria, Peoria, Illinois, United States of America; 2 Department of Pathology, University of Illinois College of Medicine at Peoria, Peoria, Illinois, United States of America; 3 Department of Neurosurgery, University of Illinois College of Medicine at Peoria, Peoria, Illinois, United States of America; University of Birmingham, United Kingdom

## Abstract

**Background:**

Glioma is the most commonly diagnosed primary brain tumor and is characterized by invasive and infiltrative behavior. uPAR and cathepsin B are known to be overexpressed in high-grade gliomas and are strongly correlated with invasive cancer phenotypes.

**Methodology/Principal Findings:**

In the present study, we observed that simultaneous downregulation of uPAR and cathepsin B induces upregulation of some pro-apoptotic genes and suppression of anti-apoptotic genes in human glioma cells. uPAR and cathepsin B (pCU)-downregulated cells exhibited decreases in the Bcl-2/Bax ratio and initiated the collapse of mitochondrial membrane potential. We also observed that the broad caspase inhibitor, Z-Asp-2, 6-dichlorobenzoylmethylketone rescued pCU-induced apoptosis in U251 cells but not in 5310 cells. Immunoblot analysis of caspase-9 immunoprecipitates for Apaf-1 showed that uPAR and cathepsin B knockdown activated apoptosome complex formation in U251 cells. Downregulation of uPAR and cathepsin B also retarded nuclear translocation and interfered with DNA binding activity of CREB in both U251 and 5310 cells. Further western blotting analysis demonstrated that downregulation of uPAR and cathepsin B significantly decreased expression of the signaling molecules p-PDGFR-β, p-PI3K and p-Akt. An increase in the number of TUNEL-positive cells, increased Bax expression, and decreased Bcl-2 expression in nude mice brain tumor sections and brain tissue lysates confirm our *in vitro* results.

**Conclusions/Significance:**

In conclusion, RNAi-mediated downregulation of uPAR and cathepsin B initiates caspase-dependent mitochondrial apoptosis in U251 cells and caspase-independent mitochondrial apoptosis in 5310 cells. Thus, targeting uPAR and cathepsin B-mediated signaling using siRNA may serve as a novel therapeutic strategy for the treatment of gliomas.

The article "Downregulation of uPAR and Cathepsin B Induces Apoptosis via Regulation of Bcl-2 and Bax and Inhibition of the PI3K/Akt Pathway in Gliomas" was retracted in 2020. Reasons: fabricated or falsified data; an official misconduct investigation; misconduct by an author; duplicated images.

## Introduction

Apoptosis is a tightly regulated form of programmed cell death involving a series of biochemical events that leads to a variety of morphological changes including membrane blebbing, cell shrinkage, nuclear fragmentation, chromatin condensation, and chromosomal DNA fragmentation [1], [2]. The components of the apoptotic signaling network are genetically encoded in an inactive form and are activated by various external and internal stimuli including DNA damage, drugs, or irradiation [3], [4]. Mitochondria play a central part in cellular survival and apoptotic death [5]. The key events of mitochondrial apoptosis include the release of cytochrome C, loss of mitochondrial transmembrane potential, altered cellular oxidation-reduction, and participation of pro- and anti-apoptotic Bcl-2 family proteins [6].

The Bcl-2 family of genes is known to be involved in the regulation of the cell death process [7], [8]. Bcl-2 and Bcl-xL are anti-apoptotic members predominantly localized in mitochondria that regulate mitochondrial membrane integrity and cytochrome C release. Pro-apoptotic members, such as Bax (Bcl-2–associated X protein) and BAD (Bcl-2-associated death promoter), mainly reside in the cytoplasm and redistribute into mitochondria in response to death stimuli [6], [9]–[11]. Bcl-2 family proteins are able to undergo homodimerization and heterodimerization, and the ratio of pro- to anti-apoptotic proteins determines the fate of cells [12], [13]. The hallmark of glioma is increased activity of the PI3K/Akt pathway that controls the expression of pro-survival proteins, including NF-κB (nuclear factor-kappaB), CREB (cAMP response element binding) (CREB) and Bcl-2 as well as pro-apoptotic molecules such as Bax and BAD [14]–[18]. CREB plays a key role in regulating neuronal survival and differentiation [19], and it promotes a pro-survival effect by regulating the transcription of several pro-survival factors, including Bcl-2 [20], [21]. In addition, in some populations of neurons, the loss of CREB imparts a Bax-dependent form of apoptosis [22].

In the present study, we demonstrate for the first time that either individual or simultaneous downregulation of uPAR and cathepsin B using siRNA decreased Bcl-2 expression and increased Bax expression in U251 glioma cells and 5310 glioma xenograft cells (*in vitro*), and in brain tumor tissue sections and tissue lysates (*in vivo*). We also show that the broad caspase inhibitor, Z-Asp-2, 6-dichlorobenzoylmethylketone rescued apoptosis in pCU-treated U251 cells, but not in 5310 cells. In addition, uPAR and cathepsin B downregulation decreased the expression levels of PDGFR-β, PI3K, and Akt and also affected the promoter (DNA) binding activity of CREB. Moreover, CREB siRNA decreased the expression of Bcl-2, but it did not affect the expression of Bax. In the present study, we also observed that PDGFR tyrosine kinase inhibitor IV decreased the expression of p-PDGFR-β and p-PI3K. Both PDGFR tyrosine kinase inhibitor IV and a PI3K inhibitor (Wortmannin) decreased the expression of p-Akt, pCREB, and Bcl-2 while increasing the expression of Bax. Taken together, the findings of the present study suggest a novel mechanism underlying uPAR and cathepsin B-mediated regulation of Bcl-2 and Bax in gliomas.

The article "Downregulation of uPAR and Cathepsin B Induces Apoptosis via Regulation of Bcl-2 and Bax and Inhibition of the PI3K/Akt Pathway in Gliomas" was retracted in 2020. Reasons: fabricated or falsified data; an official misconduct investigation; misconduct by an author; duplicated images.

## Results

### Downregulation of uPAR and cathepsin B induces apoptosis by collapsing mitochondrial membrane potential

To gain insight into the molecular roles of uPAR and cathepsin B, we knocked down the expression of these molecules using siRNA in U251 and 5310 glioma cells and then analyzed the effect on apoptosis. Western blot analysis showed that uPAR and cathepsin B expression was significantly decreased with pU, pC and pCU (Figs. 1A–B). Quantification of protein bands revealed that uPAR expression decreased by 88% in U251 cells and 68% in 5310 cells with pU (*p*<0.01). Similarly, cathepsin B expression was reduced by 76% in both cell lines when treated with pC (*p*<0.01). Cells treated with pU did not show appreciable difference in cathespin B expression as compared to controls. Similarly, cells treated with pC did not show any significant difference in expression of uPAR as compared to controls (90%). pCU-treated cells showed 95% decreased expression of uPAR in both U251 and 5310 cells. Cathepsin B expression in pCU-treated cells was significantly reduced by 90% (Fig. 1C). Immunoblot analysis for GAPDH expression revealed equal loading. Analysis of apoptotic cell distribution by FACS analysis showed that silencing of uPAR and cathepsin B expression significantly increased the apoptotic cell population in both U251 and 5310 cells (Fig. 1D). Cell cycle distribution in histograms showed that the percentage of apoptotic cell population was 2.8% in untreated U251 cells, 2.2% in SV-treated U251 cells, 70% in pU-treated U251 cells, 61% in pC-treated U251 cells, 79% in pCU-treated U251 cells, 2.5% in untreated 5310 cells, 3.0% in SV-treated 5310 cells, 72% in pU-treated 5310 cells, 65% in pC-treated 5310 cells, and 76% in pCU-treated 5310 cells (Fig. 1E).

**Figure 1:** RNAi-mediated depletion of cathepsin B and uPAR induces mitochondrial apoptosis in U251 and 5310 cells. (A–B) Western blot analysis of uPAR and cathepsin B expression in U251 and 5310 cells 72 hrs after transfection with SV, pU, pC and pCU. (C) Quantitative analysis of uPAR and cathepsin B expression by densitometry. Results from three independent experiments are shown as mean ± SD (**p<0.001). GAPDH was used as a loading control. (D) Cell cycle distribution of U251 and 5310 cells. Propidium iodide-stained cells were analyzed for DNA content using flow cytometry. (E) Histograms represent the percentage of cells in G0/G1, S and G2/M phases. The data represent one of three independent experiments. Values are mean ± SD of three different experiments (**p<0.001). (F) Cells were stained for apoptosis using TdT-mediated dUTP nick end-labeling (TUNEL) assay. Data shown are from a representative experiment. (G) Quantification of apoptotic cells expressed as percent of DAPI-stained cells. Bars represent the mean ± SD of three experiments (*p<0.05; **p<0.001). (H) Analysis of mitochondrial membrane potential using MitoLight kit. Cells were collected, incubated with MitoLight dye for 20 min at room temperature, and observed for fluorescence; red fluorescence indicates healthy cells while green fluorescence indicates apoptotic cells.

The article "Downregulation of uPAR and Cathepsin B Induces Apoptosis via Regulation of Bcl-2 and Bax and Inhibition of the PI3K/Akt Pathway in Gliomas" was retracted in 2020. Reasons: fabricated or falsified data; an official misconduct investigation; misconduct by an author; duplicated images.

In addition, TUNEL assay results for cells at 72 hrs post-transfection indicated a significant increase in TUNEL-positive cells in both U251 and 5310 cells (Fig. 1F). Quantification of apoptotic cells revealed that in 5% untreated, 6% SV-treated, 30% pU-treated, 25% pC-treated, and 58% pCU-treated U251 cells were apoptotic. 5% untreated, 6% SV-treated, 48% pU-treated, 38% pC-treated, and 64% pCU-treated 5310 cells were apoptotic as compared to DAPI stained cells (100%)(Fig. 1G). DNA fragmentation in treated samples further confirmed apoptosis (Supplementary Fig. S1). Analysis of mitochondrial membrane potential collapse by fluorescence microscopy using MitoLight dye indicated that pU, pC and pCU caused significant loss of mitochondrial membrane potential (Δψm) as indicated by a decrease in red fluorescence as compared to controls (Fig. 1H). Taken together, the data indicate that uPAR and cathepsin B play pivotal roles as anti-apoptotic molecules in glioma, and targeting uPAR and cathepsin B activity led to the induction of apoptosis.

### RNAi-mediated downregulation of uPAR and cathepsin B increases the expression of pro-apoptotic genes and decreases the expression of anti-apoptotic genes

To evaluate the expression of apoptosis-related proteins, SV- and pCU-transfected U251 and 5310 cell lysates were analyzed using RayBio Human Apoptosis Antibody Array kit. A comparison of pCU- and SV-transfected cells indicated that expression of Bax, caspase-3 and p27 increased while expression of Bcl-2 decreased with pCU in U251 cells. In pCU-treated 5310 cells, the expression of BAX increased while Bcl-2 decreased (Fig. 2A). Quantification of protein signals by densitometry revealed that both BAX and capsase-3 increased 2.5-fold and p27 increased 5.4-fold. In contrast, Bcl-2 decreased 8.6-fold in pCU-treated U251 cells. In pCU-treated 5310 cells, Bax increased 3.6-fold; however, Bcl-2 decreased 3.8-fold (Fig. 2B). To confirm these results, we determined the expression of Bcl-2 and Bax by western blot analysis using antibodies specific to Bcl-2 and Bax. The results showed that the expression of Bcl-2 was significantly decreased with pU, pC, and pCU in both U251 and 5310 cells. In contrast, expression of Bax significantly increased with these treatments (Fig. 2C). Densitometric analysis reveals that the Bcl-2/Bax ratio decreased by 65% with pU, 60% with pC, 75% with pCU in U251 as compared to controls. Similarly, in 5310 cells, the Bcl-2/Bax ratio decreased by 85% with pU, 80% with pC, and 90% with pCU as compared to controls (Fig. 2D). To determine whether decreased Bcl-2 expression and increased Bax expression were caused by gene transcription, we examined the transcript levels of Bcl-2 and Bax using semi-quantitative RT-PCR. The results show that expression of Bcl-2 mRNA was significantly decreased by pU, pC, and pCU in both U251 and 5310 cells (Fig. 2E). Furthermore, quantification by densitometry revealed that the Bcl-2/Bax ratio (at the mRNA level) decreased by 80%, 85%, and 90% with pU-, pC- and pCU-treatments. The results were similar in both U251 and 5310 cells compared to the controls (Fig. 2F).

The article "Downregulation of uPAR and Cathepsin B Induces Apoptosis via Regulation of Bcl-2 and Bax and Inhibition of the PI3K/Akt Pathway in Gliomas" was retracted in 2020. Reasons: fabricated or falsified data; an official misconduct investigation; misconduct by an author; duplicated images.

**Figure 2:** Effect of uPAR and cathepsin B downregulation on the expression of pro- and anti-apoptotic molecules. (A) Expression of pro- and anti-apoptotic molecules in U251 and 5310 cells 72 hrs after transfection with SV or pCU. Human apoptosis antibody arrays were exposed to cell lysates and processed as per the manufacturer's instructions. (B) Densitometric analysis and graphical representation of fold change of pro- and anti-apoptotic molecules. (C) Western blot analysis of Bcl-2 and Bax expression in U251 and 5310 cells 72 hrs transfection. The blots were stripped and re-probed with GAPDH antibody to verify equal loading. The experiments were repeated three times and representative blots are shown. (D) Densitometric analysis showing the Bcl-2/Bax ratio in U251 and 5310 cells. Columns: mean of triplicate experiments; bars: SE; **p<0.001. (E) Semi-quantitative RT-PCR analysis of Bcl-2 and Bax mRNA expression in pU-, pC- and pCU-transfected U251 and 5310 cells. Total RNA was extracted 72 hrs after transfection, and cDNA was synthesized as described in Materials and Methods. PCR was set up using first-strand cDNA as the template for Bcl-2, Bax and GAPDH. (F) Densitometric analysis showing the Bcl-2/Bax mRNA ratio. Columns: mean of triplicate experiments; bars: SE; **p<0.001, significant difference from untreated control or SV-transfected control.

The article "Downregulation of uPAR and Cathepsin B Induces Apoptosis via Regulation of Bcl-2 and Bax and Inhibition of the PI3K/Akt Pathway in Gliomas" was retracted in 2020. Reasons: fabricated or falsified data; an official misconduct investigation; misconduct by an author; duplicated images.

### Caspase dependent and independent apoptosis

To reveal the involvement of caspases, we used a broader caspase inhibitor, Z-Asp-2, 6-dichlorobenzoyloxymethylketone, to examine its ability to prevent apoptosis caused by uPAR and cathepsin B gene silencing. Analysis of cell distribution by FACS showed that pretreatment with the broad caspase inhibitor at 40 µM rescued the apoptosis in pCU-transfected U251 cells, but failed to prevent apoptosis in 5310 cells (Fig. 3A). Cell cycle distribution in histogram showed that the percentage of apoptotic cell population (G0–G1) was 4% in untreated, 5% in SV-treated, and 13% in pCU-treated U251 cells; in contrast, the apoptotic population was 7% in pCU-transfected cells pretreated with the broad caspase inhibitor. In 5310 cells, the percentage of the apoptotic cell population was 4% and 6% in untreated and SV-transfected cells, respectively. However, the percentage of the apoptotic cell population was 27% in both pCU-transfected cells and pCU-transfected cells pretreated with the broad caspase inhibitor (Fig. 3B). The above results indicate caspase-dependent apoptosis in U251 cells and caspase-independent apoptosis in 5310 cells.

**Figure 3:** Downregulation of uPAR and cathepsin B induced caspase-dependent apoptosis in U251 cells and caspase-independent apoptosis in 5310 cells. (A) FACS analysis of pCU-transfected U251 and 5310 cells pretreated with 40 µM broad caspase inhibitor (Z-Asp-2, 6-dichlorobenzoylmethylketone). (B) Histograms represent the percentage of cells in G0/G1, S and G2/M phases. The data represent one of the three independent experiments. Values are mean ± SD of three different experiments (*p<0.05, **p<0.001). uPAR and cathepsin B downregulation induced activation of caspase-9, caspase-3, ICAD, CAD in pU-, pC- and pCU-treated U251 cells. (C) Western blot analysis for active caspase-9, caspase-3, ICAD and CAD in U251 cells. (D) Expression of cytochrome c in mitochondrial and cytosolic fractions was determined by western blot analysis. Cytochrome oxidase IV was used as a marker for mitochondrial fractions (MF); GAPDH was used for cytosolic fractions (CF). (E) Immunoprecipitation of Apaf-1 from U251 cell lysates. Total cell lysates were subjected to immunoprecipitation using anti-caspase-9 antibody and then immunoblotted for Apaf-1. Total lysates from SV-, pU-, pC- and pCU-treated U251 cells were separated into mitochondrial and nuclear fractions as per standard protocols and immunoblotted for AIF. (F) Expression levels of AIF in mitochondrial (MF) and nuclear fractions (NF) were determined by western blot analysis. Cytochrome oxidase IV was used as a marker for mitochondrial fractions; laminin B was used for nuclear fractions. Total lysates from SV-, pU-, pC- and pCU-treated 5310 cells were fractionated into mitochondrial and cytosolic fractions as per standard protocols and immunoblotted for cytochrome c. Immunoblots are representative of three experiments.

The article "Downregulation of uPAR and Cathepsin B Induces Apoptosis via Regulation of Bcl-2 and Bax and Inhibition of the PI3K/Akt Pathway in Gliomas" was retracted in 2020. Reasons: fabricated or falsified data; an official misconduct investigation; misconduct by an author; duplicated images.

### Downregulation of uPAR and cathepsin B induces release of cytochrome c from mitochondria into cytosol and activation of caspase-3, caspase-9 and CAD in U251 cells

We performed a colorimetric assay for caspase activity in uPAR and cathepsin B siRNA-induced apoptosis in U251 cells to explore the roles of activated caspase-3 and caspase-9. We observed substantial increases in the activity of caspase-3 and caspase-9 with pU and pC and a significant increase with pCU when compared to controls (Supplementary 2). These results were confirmed by western blot analysis. Figure 3C shows that pU and pC resulted in the substantial cleavage of caspase-3, caspase-9 and CAD as compared to controls. Notably, pCU significantly increased cleaved caspase-3, caspase-9 and CAD. The cleavage of caspases is aided by the release of caspase-activating factors, particularly cytochrome c, from the mitochondrial membrane into the cytosol [23]. Hence, we determined cytochrome c levels in both mitochondrial and cytosolic fractions using western blot analysis. In the present study, we found significantly increased signal for cytochrome c in the cytosolic fractions of pU-, pC- and pCU-treated U251 cells as compared to controls. In contrast, a decreased signal for cytochrome c was noticed in mitochondrial fractions (Fig. 3D). Once released into the cytosol, cytochrome c activates apoptotic protease-activating factor (Apaf-1), which together with caspase-9, forms an active holoenzyme complex known as apoptosome [23]. To test whether uPAR and cathepsin B knockdown interferes with the formation of apoptosome complex, we performed immunoprecipitation of caspase-9 with anti-caspase-9 antibody, followed by immunoblot analysis with anti-Apaf-1 antibody. The results indicate that Apaf-1 was significantly immunoprecipitated with caspase-9 in pU-, pC- and pCU-treated samples as compared to controls (Fig. 3E).

### Downregulation of uPAR and cathepsin B activates the nuclear translocation of apoptosis-inducing factor (AIF) in 5310 glioma xenograft cells

To determine the nuclear localization of AIF, the expression levels of AIF were determined by western blot analysis of the cytoplasmic, mitochondrial and nuclear extracts of untreated and treated 5310 cells. From the results, we observed that AIF levels were remain same in the cytoplasmic extract of all treatments (data not shown). AIF levels were decreased in mitochondrial fractions of pU, pC and pCU treated 5310cells. However, nuclear localization of AIF was increased significantly when uPAR and cathepsin B were downregulated either individually or simultaneously (Fig. 3F).

The article "Downregulation of uPAR and Cathepsin B Induces Apoptosis via Regulation of Bcl-2 and Bax and Inhibition of the PI3K/Akt Pathway in Gliomas" was retracted in 2020. Reasons: fabricated or falsified data; an official misconduct investigation; misconduct by an author; duplicated images.

### Downregulation of uPAR and cathepsin B through siRNA treatment interferes with intracellular signaling events

To further elucidate uPAR and cathepsin B-mediated molecular signaling in the regulation of Bcl-2 and Bax expression, we investigated the involvement of the PI3K/Akt pathway by western blot analysis. Total PI3K (data not shown) and Akt expression levels remained more or less unchanged whereas the levels of p-PI3K p85α (Y 508) and p-Akt (S473) were significantly decreased with pCU transfection in both U251 and 5310 cells (Figs. 4A–B). Activation of PDGFR-β has been shown to induce the activation of PI3K and mediate uPA/uPAR signaling, so we next investigated the hypothesis that PDGFR-β serves as the accessory transmembrane adaptor molecule of uPAR [24]. Figures 4A–B show that expression of total PDGFR-β remained unchanged in both U251 and 5310, cells but p-PDGFR-β (Y751) significantly decreased with pCU transfection. To confirm these results, we used PI3K inhibitor (Wortmannin) at 20 and 40 µg/mL and PDGFR tyrosine kinase inhibitor (PTKI) at 5 and 10 nM concentrations. At a concentration of 40 µg/mL, the specific inhibitor of PI3K significantly inhibited basal expression of p-Akt, p-CREB (S133) and Bcl-2 and induced the expression of Bax in both U251 and 5310 cells (Figs. 4C&D). At a concentration of 10 nM, PDGFR tyrosine kinase inhibitor IV significantly inhibited the expression of p-PDGFR-β, p-PI3K, p-Akt, p-CREB and Bcl-2 and increased the expression of Bax (Figs. 4E&F).

**Figure 4:** Downregulation of uPAR and cathepsin B using siRNA interferes with intracellular signaling events. U251 and 5310 cells were transfected with SV, pU, pC or pCU. Untreated cells served as the control. After 72 hrs, cells were collected, and total cell lysates were prepared and western blotted as per standard protocol using normal and phosphorylated forms of PI3K, Akt and PDGFR-β. (A–B) Expression of normal and phosphorylated forms of PI3K, Akt and PDGFR-β in U251 and 5310 cells. Columns: mean of triplicate experiments; bars: SE; *p<005 and **p<0.001, significant difference from untreated control or SV-transfected control. Effect of PI3K inhibitor (Wortmannin) and PDGFR tyrosine kinase inhibitor (PTKI) on expression of p-PDGFR-β, p-PI3K p85α, Bcl-2 and Bax. U251 and 5310 cells were treated with 20 and 40 µg/mL of PI3K inhibitor (Wortmannin;WN) for 48 hrs, and the expression levels of p-Akt, p-CREB, Bcl-2 and Bax were determined by western blotting using appropriate antibodies. (C–D) Western blot analysis of p-AKT, p-CREB, Bcl-2 and Bax expression levels after treatment with the PI3K inhibitor. Separately, U251 and 5310 cells were treated with 5 nM and 10 nM PDGFR tyrosine kinase inhibitor (PTKI) for 48 hrs. Expression levels of p-PDGFR-β, p-PI3K, p-Akt, p-CREB, Bcl-2 and Bax were determined by western blotting using appropriate antibodies. (E–F) Western blot analysis of p-PDGFR-β, p-PI3K, p-Akt, p-CREB, Bcl-2 and Bax expression levels in U251 and 5310 cells treated with PDGFR tyrosine kinase inhibitor.

The article "Downregulation of uPAR and Cathepsin B Induces Apoptosis via Regulation of Bcl-2 and Bax and Inhibition of the PI3K/Akt Pathway in Gliomas" was retracted in 2020. Reasons: fabricated or falsified data; an official misconduct investigation; misconduct by an author; duplicated images.

### uPAR and cathepsin B downregulation retards nuclear translocation and affects DNA binding activity of CREB

It has been shown that Bcl-2 expression might be regulated by the transcription factor CREB [25], so we investigated expression and phosphorylation of CREB in nuclear extracts of U251 and 5310 cells using western blotting. The results depicted in Figures 5A–B show that expression of total CREB was not altered; however expression of p-CREB was significantly decreased in the nuclear fraction of pCU-transfected U251 and 5310 cells as compared to controls. To further investigate the effect of uPAR and cathepsin B downregulation on CRE binding activity of CREB, we used antibody induced supershift analysis in EMSA. Nuclear extracts from SV- and pCU- treated cells showed supershift with strong binding when subjected to antibody induced supershift in EMSA. However, the intensity of the band showing supershift in pCU-treated cells was significantly decreased (Figs. 5C–D, lane 5). In contrast, with either no antibody or normal IgG antibody the CREB DNA binding mobility was not affected (Figs. 5C–D, lanes1, 3, 4 and 6). Taken together, these results strongly support that pCU-treatment specifically decreased the DNA binding activity of CREB.

**Figure 5:** uPAR and cathepsin B downregulation retards nuclear translocation and decreases DNA binding activity of CREB. U251 and 5301 cells were transfected with SV, pU, pC or pCU for 72 hrs. Cell lysates were separated into nuclear (NF) and cytoplasmic fractions (CF) and immunoblotted for p-CREB. Total cell lysates were probed for CREB. (A–B) Western blot analysis of p-CREB in nuclear and cytoplasmic fractions of U251 and 5310 cells. Nuclear extracts were prepared from SV- (control) and pCU-transfected U251 and 5310 cells and supershift analysis of CREB binding activity was carried out using EMSA. For supershift analysis, nuclear extracts were incubated with supershift specific CREB antibody (2.0 µg) or IgG (2.0 µg) prior to incubation with CREB binding buffer. (C–D) Supershift analysis of CREB DNA binding activity in U251 and 5310 cells. The experiments were performed three times and representative blots are shown. Nuclear extracts were prepared from SV-, pU-, pC- and pCU-transfected U251 and 5310 cells, and DNA binding activity of CREB was determined by colorimetric assay using the TransAM ELISA kit. To test specificity, DNA binding activity was tested in the presence of an excess of oligonucleotide containing a wild-type or mutated CREB consensus binding site. (E–F) Inhibition of DNA binding activity of CREB by nuclear extracts of pU-, pC- and pCU-treated U251 and 5310 cells. The bars represent the mean ± SD of three different experiments. *Statistically different compared to controls and pU-, pU- and pCU-treated groups (**p<0.001).

The article "Downregulation of uPAR and Cathepsin B Induces Apoptosis via Regulation of Bcl-2 and Bax and Inhibition of the PI3K/Akt Pathway in Gliomas" was retracted in 2020. Reasons: fabricated or falsified data; an official misconduct investigation; misconduct by an author; duplicated images.

DNA-binding activity of CREB was also determined by colorimetric assay using the TransAM ELISA kit. To test the specificity of DNA binding, the assay was also performed in the presence of excess oligonucleotide containing a wild-type or mutated CREB consensus binding site. At 20X excess, the wild-type oligonucleotide prevents CREB binding to the probe immobilized on the plate. Conversely, the mutated oligonucleotide has little effect on CREB binding. The results show that without probe, optical density (OD) at 450 nm was 2.55 in nuclear extracts of untreated U251 and 5310 cells (control). In contrast, the OD was 1.25 in both pU- and pC-treated nuclear extracts of U251 cells and 1.3 and 1.5 in pU- and pC-treated nuclear extracts of 5310 cells. However, OD of all nuclear extracts with wild-type and mutated consensus oligonucleotides was 3, which indicates specific binding of CREB with CREB responsive elements (Figs. 5E–F). To further confirm CREB-mediated regulation of Bcl-2 and Bax, we treated both U251 and 5310 cells with CREB siRNA for 48 hrs and determined the expression of CREB, Bcl-2 and Bax using western blotting. The results indicate that expression levels of CREB and Bcl-2 were significantly decreased with CREB gene silencing in both U251 and 5310 cells. However, expression of BAX remains same in controls and siRNA treated U251 and 5310 cells (Supplementary Fig. S3).

### pCU induces apoptosis, inhibits expression of uPAR, cathepsin B and Bcl-2, and enhances expression of BAX *in vivo*

To correlate the *in vitro* results with *in vivo* experiments, we further investigated the effect of uPAR and cathepsin B downregualtion on apoptosis using U251 and 5310 cells in nude mice. After the mice were implanted with U251 and 5310 cells as explained in Materials and Methods, the mice were observed for 30 days. Tumor samples were then taken and paraffin-embeded sections were prepared for immunohistopathological examination. These *in vivo* experiments would be helpful to confirm our *in vitro* data showing that uPAR and cathepsin B downregulation induces apoptosis in the glioma cells. To check the apoptosis in *in vivo*, we have carried out TUNEL assay on paraffin-embedded brain tissue sections. The results demonstrated significant DNA fragmentation in pCU-treated brain tissue sections as compared to control sections (Figs. 6A–B). Next, we determined expression of uPAR, cathepsin B, Bcl-2 and Bax in brain tissue lysates and tissue sections. Immunohistochemical analysis revealed that expression levels of uPAR, cathepsin B and Bcl-2 were decreased in pCU-treated brain tissue sections of both U251 and 5310 as compared to controls. In contrast, expression of Bax was increased in pCU-treated brain tissue sections as compared to controls (Figs. 6C–D). Western blot analysis further confirmed that pCU significantly inhibited the expression of uPAR, cathepsin B and Bcl-2 while the expression of BAX increased in both U251 and 5310 brain tissue lysates as compared to controls (Figs. 6E–F).

The article "Downregulation of uPAR and Cathepsin B Induces Apoptosis via Regulation of Bcl-2 and Bax and Inhibition of the PI3K/Akt Pathway in Gliomas" was retracted in 2020. Reasons: fabricated or falsified data; an official misconduct investigation; misconduct by an author; duplicated images.

**Figure 6:** RNAi-mediated downregulation of uPAR and cathepsin B induces apoptosis in pre-established intracranial tumors. Intracranial tumors were established in nude mice by injecting U251 and 5310 cells that were treated with SV and pCU as described in Materials and Methods. (A–B) The brains were embedded in paraffin, sectioned and stained for apoptosis by TdT-mediated nick end-labeling (TUNEL) followed by DAB staining. Nuclei were counterstained with methyl green. Data shown are representative of five fields. Brown stain around green nuclei indicates apoptotic cells. (C–D) Immunohistochemical analysis of uPAR, cathepsin B, Bcl-2 and Bax was performed in paraffin-embedded U251 and 5310 tumor sections. Appropriate protein-specific antibodies were used. Fields with brown staining as a result of DAB interaction were scored for protein expression. (E–F) uPAR and cathepsin B, Bcl-2 and Bax expression was detected in tumor tissue lysates from intracranial tumors of mice that received SV and pCU. Results are representative of three separate experiments.

## Discussion

uPAR and cathepsin B are overexpresssed in high-grade glioma, and this overexpression strongly correlates with invasive cancer phenotype and poor prognosis [26]–[29]. As stated earlier, RNAi has emerged as potent technology for exploiting target genes in glioma. As a preliminary assessment of the potential of RNAi against uPAR and cathepsin B as a therapeutic agent in growth inhibition, we assessed its *in vitro* apoptotic activity against U251 glioma and 5310 glioma xenograft cells. Transfection of glioma cells with siRNA for uPAR and/or cathepsin B strongly inhibited the expression of both proteins as previously reported [30]. When glioma cells were transfected with the bicistronic construct pCU, the morphology of cells became rounded and growth was inhibited (data not shown), which is suggestive of apoptosis. Further, our investigation using flow cytometric analysis and TUNEL assay confirmed that cell death induced by pU, pC and pCU transfection was due to induction of apoptosis.

The article "Downregulation of uPAR and Cathepsin B Induces Apoptosis via Regulation of Bcl-2 and Bax and Inhibition of the PI3K/Akt Pathway in Gliomas" was retracted in 2020. Reasons: fabricated or falsified data; an official misconduct investigation; misconduct by an author; duplicated images.

Mitochondria are the central integrators and coordinators of both intracelluar and extracellular signals that mediate caspase-dependent and caspase-independent cell death [31]. Recently, it has been reported that induction of mitochondrial apoptosis requires the involvement of the Bcl-2 family, including apoptosis inhibiting gene products (*e.g.*, Bcl-2, Bcl-xL) and apoptosis accelerating gene products (e.g., Bax, Bak, Bcl-xS, Bim) [32]. Loss of mitochondrial membrane potential is a prerequisite for mitochondrial-mediated apoptosis as it is associated with the reshuffling of Bcl-2 family members between the cytoplasm and mitochondria. The Bcl-2 family is comprised of proteins, which share a Bcl-2 homology (BH) region and undergo either heterodimerization or homodimerizaton [33]. The ratio between anti- and pro-apoptotic proteins is said to be a determinant for tissue homeostasis because it influences the sensitivity of cells to inducers of apoptosis [34], [35]. Overexpression of Bcl-2 is reported to cause inhibition of programmed cell death in many cell types, and this anti-apoptotic function appears to be modulated by its ability to heterodimerize with other members of the family, especially the apoptosis-inducing Bax protein [36].

In this study, we have demonstrated that the downregulation of uPAR and cathepsin B induced mitochondrial-mediated apoptosis in the U251 glioma cell line and 5310 glioma xenograft cells and was accompanied by the collapse of mitochondrial membrane potential. We also noticed that downregulation of uPAR and cathepsin B decreased the Bcl-2/Bax ratio. An earlier study reported that downregulation of uPAR and cathepsin B initiated partial extrinsic apoptotic cascade accompanied by the collapse of mitochondrial membrane potential in SNB19 glioma cells [37]. Moreover, Kin et al. [38] reported that downregulation of uPAR was associated with increased expression of the pro-apoptotic protein Bax in glioma cells. Taken together, these results suggest that uPAR and cathepsin B downregulation induced apoptosis by modulating the Bcl-2/Bax ratio accompanied by collapse of mitochondrial membrane potential.

The article "Downregulation of uPAR and Cathepsin B Induces Apoptosis via Regulation of Bcl-2 and Bax and Inhibition of the PI3K/Akt Pathway in Gliomas" was retracted in 2020. Reasons: fabricated or falsified data; an official misconduct investigation; misconduct by an author; duplicated images.

In the present study, significant increases in caspase-3, Apaf-1 and cytochrome c were also observed with the downregulation of uPAR and cathepsin B in U251 cells but not in 5310 cells (data not shown). In contrast, in 5310 cells, the downregulation of uPAR and cathepsin B was accompanied by the nuclear translocation of AIF from the mitochondria. Cytochrome c combines with Apaf-1, caspase-9 and ATP to form the apoptosome in the cytoplasm [39]. AIF is another mitochondrial protein that is translocated to the cytosol and nucleus during apoptosis [40]. In the nucleus, AIF is thought to increase chromatin condensation and large-scale DNA fragmentation [41]. Interestingly, a broad caspase inhibitor, Z-Asp-2-6-dichlorobenzoylmethylketone, prevented pCU-induced apoptosis in U251 cells but fail to reduce the apoptotic percentage of 5310 xenograft cells, which indicates caspase-dependent apoptosis in U251 cells and caspase-independent apoptosis in 5310 cells. Similarly, Shih et al. [42] reported that cadmium induced a caspase-independent apoptotic pathway involving mitochondria-mediated translocation of AIF in normal human lung cells. Further, Tae-Jin Lee et al. [43] also reported caspase-dependent and caspase-independent apoptosis in human leukemic U937 cells.

The translocation of AIF and release of cytochrome c would occur after the collapse of mitochondrial membrane potential. However, mechanisms of membrane permeabilization are still matter of debate. Irrespective of the exact mechanisms, the anti-apoptotic members of the Bcl-2 family tend to stabilize the barrier function of mitochondrial membranes, whereas pro-apoptotic Bcl-2 family proteins destabilize it [44]. uPAR is a GPI-anchored cell surface protein known to be associated with pro-uPA and cathepsin B [45]. uPAR relies on cell surface and transmembrane proteins, including platelet-derived growth factor receptor (PDGFR) for its non-proteolytic functions [46]. Recently, a direct interaction of uPAR with PDGFR beta in macrophages [24] and vascular smooth muscle cells [44] by the immunefluorescence approach, immunoprecipitation and chemical cross linking experiments have been reported. Further, the effect of cathepsin B on PDGFR beta mediated signaling might be indirect and possibly through uPAR.

In the current study, western blot analysis using phospho-specific antibodies confirmed that expression of p-PDGFR-β, p-PI3K and p-Akt were significantly decreased with the downregulation of uPAR and cathepsin B in both U251 and 5310 cells. However, this protein phosphorylation was inhibited by pre-treatment with PDGFR tyrosine kinase inhibitor IV and PI3K inhibitor. It is well known that tyrosine kinase activity of PDGFR-β was found to be decisive for mediating downstream signaling. Duronio [47] recently reported that PDGFR-β is associated with PI3K/Akt-mediated cell survival. These results further confirm that uPAR-initiated signaling is mediated though PDGFR-β and the PI3K/Akt pathway.

The article "Downregulation of uPAR and Cathepsin B Induces Apoptosis via Regulation of Bcl-2 and Bax and Inhibition of the PI3K/Akt Pathway in Gliomas" was retracted in 2020. Reasons: fabricated or falsified data; an official misconduct investigation; misconduct by an author; duplicated images.

Recently, CREB was reported to be activated as a transcription factor by phosphorylation at Ser-133 through several signaling pathways, including PI3K/Akt [48]. Pugazhenthi et al. [49] reported that Akt/protein kinase B upregulates Bcl-2 expression through cAMP-response element-binding protein. CREB plays a key role in regulating neuronal survival and appears to be a primary transcription activator of the anti-apoptotic gene, Bcl-2 [50], [51]. CREB mediates regulation of gene expression via its binding to a CRE in the promoter region [52].

In this study, western blot analysis of cytoplasmic and nuclear fractions showed that uPAR and cathepsin B downregulation retarded the translocation of p-CREB in both U251 and 5310 cells. In addition, analysis of DNA binding activity by EMSA and ELISA revealed that uPAR and cathepsin B downregulation also affected DNA binding activity of CREB. To our knowledge, this is the first report on the uPAR and cathepsin B-mediated regulation of DNA binding activity of CREB in glioma. Moreover, knockdown of CREB using siRNA significantly decreased expression of Bcl-2 but not Bax. Further, use of a PI3K inhibitor significantly decreased the expression of both Bcl-2 and Bax. These results suggest that uPAR and cathepsin B downregulation suppressed Bcl-2 expression possibly though inhibition of the PI3/Akt pathway and regulation of DNA binding activity (transcriptional) of CREB. However, Bax levels might be enhanced by retaining Bax in the cytoplasm. This is an accordance with an earlier study that reported PI3K/AKT activity was essential for retaining Bax in the cytoplasm [18].

It has been previously demonstrated that *in vivo* treatment of pre-established intracranial tumors with plasmids expressing siRNA for uPAR and cathepsin B significantly inhibited tumor growth in glioma [53]. In this study, we observed significant cell death in pCU-treated U251 and 5310 brain tissue sections. In addition, immunohistochemical analysis for Bcl-2 and Bax in tumor brain sections treated with pCU and western blot analysis of Bcl-2 and Bax in brain tissue lysates strongly confirmed our *in vitro* results. Further, simultaneous downregulation of two molecules using bicistronic vectors proved to be more effective than specifically targeting a single gene/molecule [54]. However, the mechanism of cell cycle and apoptosis is highly complex and involves coordinated regulation of several molecules. Each of these molecules might have a specific and independent role in apoptosis; hence the effect is not always synergistic [55]. Studies have also shown that the cellular proteases can either act independently or coordinate with other proteases in the process of invasion, angiogenesis and apoptosis [56], [57]. In conclusion, downregulation of uPAR and/or cathepsin B induced mitochondrial-mediated apoptosis by modulating the Bcl-2/Bax ratio via inhibition of PDGFR-β and the PI3K/Akt pathway (Fig. 7). Taken together, our results suggest uPAR and cathepsin B are promising potential therapeutic targets for glioma.

The article "Downregulation of uPAR and Cathepsin B Induces Apoptosis via Regulation of Bcl-2 and Bax and Inhibition of the PI3K/Akt Pathway in Gliomas" was retracted in 2020. Reasons: fabricated or falsified data; an official misconduct investigation; misconduct by an author; duplicated images.

**Figure 7:** Schematic representation of proposed molecular mechanisms involved in the regulation of mitochondrial-mediated apoptosis via PDGFR β and the PI3K/Akt pathway in uPAR and cathepsin B-depleted glioma cells.

## Materials and Methods

### Ethics Statement

The Institutional Animal Care and Use Committee of the University of Illinois College of Medicine at Peoria, Peoria, IL, USA approved all surgical interventions and post-operative animal care. The consent was written and approved. The approved protocol number is 851, dated November 20, 2009.

### Cell culture and transfection conditions

We used the U251 glioblastoma cancer cell line (obtained from ATCC) and 5310 glioblastoma xenograft cells (kindly provided by Dr. David James, University of California, San Francisco) in this study. U251 and 5310 cells were grown in DMEM/F12 medium and RPMI 1640 medium, respectively and supplemented with 10% FBS and 1% penicillin/streptomycin. After overnight culturing in serum-free medium, cells were transfected with scrambled vector (SV), puPAR (pU), pCathepsin B (pC), or a bicistronic construct comprised of puPAR and pCathepsin B (pCU) for 72 hrs using FuGene according to manufacturer's instructions (Roche Applied Science, IN). For CREB knockdown, U251 and 5310 cells were transfected with CREB siRNA for 48 hrs using FuGene according to manufacturer's instructions (Cell Signaling Tech., Danvers, MA).

### Western blotting and immunoprecipitation

U251 and 5310 glioma cells or brain tissues were harvested as previously described [58]. Equivalent amounts of total protein (30–50 µg per lane) were loaded onto 6–14% acrylamide gels, resolved by electrophoresis, and electrotransferred onto nitrocellulose membranes. Membranes were blocked and subsequently incubated overnight at 4°C with primary antibodies. We obtained all of the antibodies used in this study from Santa Cruz Biotechnology (Santa Cruz, CA) except for anti-PDGFR-β, anti-p-PDGFR-β, anti-Akt, anti-p-Akt, anti-PI3K, anti-p-PI3K, anti-CREB, anti-p-CREB (S133), anti-Bcl-2, and anti-Bax, which were supplied by Cell Signaling (Boston, MA). Primary antibodies were detected with horseradish peroxidase (HRP)-conjugated secondary antibody raised against the corresponding species for 1 hr at room temperature. Proteins on membranes were developed using Pierce ECL Western Blotting Substrate according to manufacturer's instructions (Thermo Scientific Inc, Rockford, IL). Protein content was normalized against the GAPDH level, which was used as a loading control.

The article "Downregulation of uPAR and Cathepsin B Induces Apoptosis via Regulation of Bcl-2 and Bax and Inhibition of the PI3K/Akt Pathway in Gliomas" was retracted in 2020. Reasons: fabricated or falsified data; an official misconduct investigation; misconduct by an author; duplicated images.

Caspase-9 was immunoprecipitated from 300 µg of total protein using anti-caspase-9 antibody and protein A coupled with G agarose beads (20 µg). The precipitates were washed five times with lysis buffer and once with PBS. The pellet was then resuspended in 1X sample buffer [50 mM Tris, (pH 6.8), 100 mM bromophenol blue, and 10% glycerol], incubated at 90°C for 10 min before electrophoresis to release the proteins from the beads, and then immunoblotted for Apaf-1.

### Cell cycle analysis

Phases of cell cycle were analyzed using flow cytometry as described previously [59]. Cells transfected with SV, pU, pC, pCU or pCU + pretreatment with broad caspase inhibitor were trypsinized, washed with 1X PBS, and incubated with 1 mL of propidium iodide for 30 min in the dark. The DNA content of these cells was measured based on the presence of propidium iodide (PI)-stained cells (Sigma Aldrich, St. Louis, MO). Flow cytometric analysis was carried out on at least 10,000 cells from each sample, and cell cycle data were analyzed using a FACS Calibur flow cytometer (BD BioSciences, San Jose, CA) with an excitation wavelength of 488 nm and an emission wavelength of 530 nm.

### TUNEL assay

TUNEL assay was performed with adherent cells [40] and paraffin-embedded tissue sections [60] using *In Situ* Cell Death Detection Kit (Roche Diagnostics Corp., Indianapolis, IL). After transfection with SV, pU, PC, or pCU, cells were fixed with buffered formaldehyde (pH 7.4) and incubated with a reaction mixture containing biotin-dUTP and terminal deoxynucleotidyl transferase for 1 hr. The slides were stained with DAPI, mounted with cover slips, and positively fluorescein-labeled cells were visualized with fluorescence microscopy, quantified, and expressed as percent compared to DAPI stained cells. For tissue sections, after deparaffinization and rehydration, tissue sections were pretreated with sodium chloride-sodium citrate buffer (pH 7.0) at 80°C for 20 min, followed by thorough washing in distilled water. Subsequently, sections were digested with Proteinase K for 1 hr with gentle agitation at 37°C and digestion was stopped by washing in running water. After protease treatment, tissue sections were treated as described above and subsequently stained with DAB via peroxidase-conjugated avidin and counterstained with 0.5% methyl green.

The article "Downregulation of uPAR and Cathepsin B Induces Apoptosis via Regulation of Bcl-2 and Bax and Inhibition of the PI3K/Akt Pathway in Gliomas" was retracted in 2020. Reasons: fabricated or falsified data; an official misconduct investigation; misconduct by an author; duplicated images.

### Visualization of mitochondrial permeability transition

Mitochondrial membrane potential changes were assayed with MitoLight dye according to manufacturer's instructions (Millipore, Danvers, MA). After transfection with SV, pU, pC or pCU, cells were incubated with pre-diluted MitoLight solution for 30 min. Cells were washed twice with 1X incubation buffer, mounted with cover slips, and observed immediately under a fluorescence microscope.

### Apoptosis array

Cell lysates from SV- and pCU-treated U251 and 5310 cells were analyzed using a human apoptosis antibody array (RayBiotech, Norcross, GA) according to the manufacturer's instructions. Signal intensities were quantified by densitometry, and fold change was calculated by comparing with controls.

### Reverse transcription PCR (RT-PCR)

Total RNA was extracted from the transfected cells using TRIZOL reagent (Invitrogen, Carlsbad, CA) as per standard protocol. DNase-treated RNA was used as a template for reverse transcription (Invitrogen) followed by PCR analysis using specific primers for Bcl-2, Bax and GAPDH (Table 1). The PCR conditions were as follows: 94°C for 5 min, followed by 35 cycles of 94°C for 30 sec, 58°C for 45 sec, and 72°C for 45 sec. GAPDH was used as an internal control.

**Table 1:** Genes analyzed by RT-PCR.

Gene	Forward Primer	Reverse Primer
Bcl-2	5′TTCCACGCCGAAGGACAGCG 3′	5′GGCACTTGTGGCGGCCTGAT 3′
BAX	5′AGTGGCAGCTGACATGTTTT 3′	5′GGAGGAAGTCCAATGTCCAG 3′
GAPDH	5′CGGAGTCAACGGATTTGGTCGTAT 3′	5′AGCCTTCTCCATGGTGGTGAAGAC3′

### DNA binding activity of CREB

The interaction of CREB protein with DNA present in the nuclear extracts from SV- and pCU-treated U251 and 5310 cells was determined by supershift analysis experiments in EMSA using Pamomics kit according to manufacturer's instructions Affymetrix Inc, Fremont, CA). Briefly, nuclear extracts were incubated with supershift specific antibody (2.0 µg) (Santa Cruz Biotechnology, SC:271x) and normal IgG antibody (2.0 µg) for 30 min prior to incubation with biotin-labeled CREB transcription probe. The protein/DNA complexes were separated on a 6% non-denaturing polyacrylamide gel, and then they were transferred to a nylon membrane and detected using streptavidin-HRP and a chemiluminescent substrate.

DNA-binding activity of CREB was confirmed by ELISA (Active Motif, which is based on multi-well plates coated with an oligonucleotide containing the consensus binding site of the transcription factor), according to the manufacturer's recommendations. Briefly, 10 µg of nuclear proteins were incubated for 2 hrs in a 96-well plate pre-coated with a double-stranded oligonucleotide containing the consensus CRE site (TGACGTCA). Specificity of binding was also determined using wild-type and mutated consensus oligonucleotides. Binding of p-CREB was determined with an anti-Ser^133^-pCREB rabbit antibody. Colorimetric reaction was then performed with a HRP-conjugated, anti-rabbit IgG antibody, and absorbance was measured at 450 nm in a spectrophotometer.

The article "Downregulation of uPAR and Cathepsin B Induces Apoptosis via Regulation of Bcl-2 and Bax and Inhibition of the PI3K/Akt Pathway in Gliomas" was retracted in 2020. Reasons: fabricated or falsified data; an official misconduct investigation; misconduct by an author; duplicated images.

### Subcellular fractionation

Fractionation of nuclear and cytosolic proteins was carried out as previously described [40]. Fractionation of mitochondrial proteins was done using a mitochondrial isolation kit (Sigma, St. Louis, MO) according to manufacturer's instructions. Briefly, cells were suspended in cell lysis buffer and homogenized on ice using a Dounce homogenizer (10–30 strokes) and centrifuged at 600×*g* for 10 min at 4°C. The supernatant was carefully transferred to a fresh tube and centrifuged at 11,000×*g* for 10 min at 4°C. The supernatant was discarded and the pellet was resuspended in CellLytic M cell lysis reagent with a protease inhibitor cocktail (1∶100 [v/v]) and used to analyze mitochondrial proteins.

### Immunohistochemical analysis of brain tumor sections for Bcl-2 and Bax

Stereotactic implantation of untreated, SV-, or pCU-treated U251 and 5310 cells (1×10^5^) was performed using Alzet minipumps at the rate of 0.25 µL/hr. Sacrifice of glioma-bearing mice and tumor processing were done as previously described [61], [62]. Five animals were used per treatment condition. Immunohistochemical analysis for Bcl-2 and Bax was performed using standard protocols.

### Caspase activity assay

The activity of caspase-3 and caspase-9 was determined using colorimetric assay according to manufacturer's instructions (Chemicon International Inc., Temecula, CA). The lysates were transferred to a 96-well plate and treated with the respective peptide substrate for each caspase conjugated with *p*-nitroaniline (Ac-DEVD-pNA). After overnight incubation, OD was measured at 405 nm using a microplate reader.

### DNA laddering assay

DNA laddering assay was carried out as described previously [63]. Briefly, untreated and treated cells were resuspended in PBS, fixed in 70% ethanol, and incubated overnight at −20°C. Ethanol was removed by centrifugation at 5000 rpm for 3 min, and the pellet was resuspended in 0.2 M phosphate-citrate buffer (pH 7.8) and kept at room temperature for 30 min. The pellet was then spun down at 10,000 rpm for 5 min, mixed with 3 µL of NP-40 and 3 µL of RNase A, and then incubated at 37°C for 30 min. After adding 3 µL of Proteinase K solution, the mixture was incubated for an additional 30 min. An aliquot of each DNA extract was then mixed with loading buffer and separated on a 1.5% agarose gel. DNA fragmentation was visualized under UV light after staining with ethidium bromide.

The article "Downregulation of uPAR and Cathepsin B Induces Apoptosis via Regulation of Bcl-2 and Bax and Inhibition of the PI3K/Akt Pathway in Gliomas" was retracted in 2020. Reasons: fabricated or falsified data; an official misconduct investigation; misconduct by an author; duplicated images.

## Supporting Information

Figure S1 RNAi-mediated downregulation of uPAR and cathepsin B induces DNA fragmentation in U251 and 5320 cells. Untreated and treated cells were fixed in 70% ethanol overnight at −20°C. Ethanol was removed, and DNA was extracted and separated on 1.5% agarose gels as described in Materials and Methods. DNA fragmentation was visualized under UV light after staining with ethidium bromide. Agarose gel electrophoresis pattern of DNA obtained from U251 and 5310 cells after transfection with SV, pU, pC or pCU. Arrow indicates 180 bp laddering.
(0.60 MB TIF)

Figure S2 RNAi-mediated downregulation of uPAR and cathepsin B enhances activity of caspase-3 and caspase-9 in U251 and 5310 cells. Cell lysates were prepared from U251 cells transfected with SV, pU, pC or pCU and treated overnight with the respective peptide substrate for each caspase conjugated with p-nitroaniline (Ac-DEVD-pNA). Activity of these proteases was measured at 405 nm using a microplate reader. Bars represent the mean ± SD of three experiments (*p<0.05, **p<0.001).
(0.03 MB TIF)

Figure S3 Effect of CREB knockdown on Bcl-2 and Bax expression. U251(A) and 5310(B) cells were transfected with CREB siRNA for 48 hrs, and the expression levels of total CREB, p-CREB, Bcl-2 and Bax were determined by western blot analysis using appropriate antibodies.
(0.14 MB TIF)

## References

[1] Huppertz B, Frank HG, Kaufmann P (1999). The apoptosis cascade–morphological and immunohistochemical methods for its visualization.. Anat Embryol (Berl).

[2] Wyllie AH, Kerr JF, Currie AR (1980). Cell death: the significance of apoptosis.. Int Rev Cytol.

[3] Giovannini C, Scazzocchio B, Vari R, Santangelo C, D'Archivio M (2007). Apoptosis in cancer and atherosclerosis: polyphenol activities.. Ann Ist Super Sanita.

[4] Ishizaki Y, Cheng L, Mudge AW, Raff MC (1995). Programmed cell death by default in embryonic cells, fibroblasts, and cancer cells.. Mol Biol Cell.

[5] Mayer B, Oberbauer R (2003). Mitochondrial regulation of apoptosis.. News Physiol Sci.

[6] Green DR, Reed JC (1998). Mitochondria and apoptosis.. Science.

[7] Adams JM, Cory S (2001). Life-or-death decisions by the Bcl-2 protein family.. Trends Biochem Sci.

[8] Adams JM, Cory S (1998). The Bcl-2 protein family: arbiters of cell survival.. Science.

[9] Gross A, McDonnell JM, Korsmeyer SJ (1999). BCL-2 family members and the mitochondria in apoptosis.. Genes Dev.

[10] Kroemer G, Reed JC (2000). Mitochondrial control of cell death.. Nat Med.

The article "Downregulation of uPAR and Cathepsin B Induces Apoptosis via Regulation of Bcl-2 and Bax and Inhibition of the PI3K/Akt Pathway in Gliomas" was retracted in 2020. Reasons: fabricated or falsified data; an official misconduct investigation; misconduct by an author; duplicated images.

[11] Vander Heiden MG, Thompson CB (1999). Bcl-2 proteins: regulators of apoptosis or of mitochondrial homeostasis?. Nat Cell Biol.

[12] Martin S, Toquet C, Oliver L, Cartron PF, Perrin P (2001). Expression of bcl-2, bax and bcl-xl in human gliomas: a re-appraisal.. J Neurooncol.

[13] Oltvai ZN, Milliman CL, Korsmeyer SJ (1993). Bcl-2 heterodimerizes in vivo with a conserved homolog, Bax, that accelerates programmed cell death.. Cell.

[14] Creson TK, Yuan P, Manji HK, Chen G (2009). Evidence for involvement of ERK, PI3K, and RSK in induction of Bcl-2 by valproate.. J Mol Neurosci.

[15] Datta SR, Dudek H, Tao X, Masters S, Fu H (1997). Akt phosphorylation of BAD couples survival signals to the cell-intrinsic death machinery.. Cell.

[16] Du K, Montminy M (1998). CREB is a regulatory target for the protein kinase Akt/PKB.. J Biol Chem.

[17] Kane LP, Shapiro VS, Stokoe D, Weiss A (1999). Induction of NF-kappaB by the Akt/PKB kinase.. Curr Biol.

[18] Tsuruta F, Masuyama N, Gotoh Y (2002). The phosphatidylinositol 3-kinase (PI3K)-Akt pathway suppresses Bax translocation to mitochondria.. J Biol Chem.

[19] Finkbeiner S, Tavazoie SF, Maloratsky A, Jacobs KM, Harris KM (1997). CREB: a major mediator of neuronal neurotrophin responses.. Neuron.

[20] Meller R, Minami M, Cameron JA, Impey S, Chen D (2005). CREB-mediated Bcl-2 protein expression after ischemic preconditioning.. J Cereb Blood Flow Metab.

[21] Riccio A, Ahn S, Davenport CM, Blendy JA, Ginty DD (1999). Mediation by a CREB family transcription factor of NGF-dependent survival of sympathetic neurons.. Science.

[22] Lonze BE, Riccio A, Cohen S, Ginty DD (2002). Apoptosis, axonal growth defects, and degeneration of peripheral neurons in mice lacking CREB.. Neuron.

[23] Lademann U, Cain K, Gyrd-Hansen M, Brown D, Peters D (2003). Diarylurea compounds inhibit caspase activation by preventing the formation of the active 700-kilodalton apoptosome complex.. Mol Cell Biol.

[24] Fuhrman B, Gantman A, Khateeb J, Volkova N, Horke S (2009). Urokinase activates macrophage PON2 gene transcription via the PI3K/ROS/MEK/SREBP-2 signalling cascade mediated by the PDGFR-beta.. Cardiovasc Res.

[25] Wilson BE, Mochon E, Boxer LM (1996). Induction of bcl-2 expression by phosphorylated CREB proteins during B-cell activation and rescue from apoptosis.. Mol Cell Biol.

[26] Gladson CL, Pijuan-Thompson V, Olman MA, Gillespie GY, Yacoub IZ (1995). Up-regulation of urokinase and urokinase receptor genes in malignant astrocytoma.. Am J Pathol.

[27] Mohanam S, Sawaya R, McCutcheon I, Ali-Osman F, Boyd D (1993). Modulation of in vitro invasion of human glioblastoma cells by urokinase-type plasminogen activator receptor antibody.. Cancer Res.

The article "Downregulation of uPAR and Cathepsin B Induces Apoptosis via Regulation of Bcl-2 and Bax and Inhibition of the PI3K/Akt Pathway in Gliomas" was retracted in 2020. Reasons: fabricated or falsified data; an official misconduct investigation; misconduct by an author; duplicated images.

[28] Sivaparvathi M, Sawaya R, Wang SW, Rayford A, Yamamoto M (1995). Overexpression and localization of cathepsin B during the progression of human gliomas.. Clin Exp Metastasis.

[29] Yamamoto M, Sawaya R, Mohanam S, Rao VH, Bruner JM (1994). Expression and localization of urokinase-type plasminogen activator receptor in human gliomas.. Cancer Res.

[30] Gondi CS, Lakka SS, Dinh DH, Olivero WC, Gujrati M (2004). RNAi-mediated inhibition of cathepsin B and uPAR leads to decreased cell invasion, angiogenesis and tumor growth in gliomas.. Oncogene.

[31] Cregan SP, Dawson VL, Slack RS (2004). Role of AIF in caspase-dependent and caspase-independent cell death.. Oncogene.

[32] Brunelle JK, Letai A (2009). Control of mitochondrial apoptosis by the Bcl-2 family.. J Cell Sci.

[33] Steinbach JP, Weller M (2004). Apoptosis in gliomas: molecular mechanisms and therapeutic implications.. J Neurooncol.

[34] Korsmeyer SJ (1999). BCL-2 gene family and the regulation of programmed cell death.. Cancer Res.

[35] Reed JC (1999). Dysregulation of apoptosis in cancer.. J Clin Oncol.

[36] Reed JC (1997). Double identity for proteins of the Bcl-2 family.. Nature.

[37] Gondi CS, Kandhukuri N, Kondraganti S, Gujrati M, Olivero WC (2006). RNA interference-mediated simultaneous down-regulation of urokinase-type plasminogen activator receptor and cathepsin B induces caspase-8-mediated apoptosis in SNB19 human glioma cells.. Mol Cancer Ther.

[38] Kin Y, Chintala SK, Go Y, Sawaya R, Mohanam S (2000). A novel role for the urokinase-type plasminogen activator receptor in apoptosis of malignant gliomas.. Int J Oncol.

[39] Hajra KM, Liu JR (2004). Apoptosome dysfunction in human cancer.. Apoptosis.

[40] Gondi CS, Talluri L, Dinh DH, Gujrati M, Rao JS (2009). RNAi-mediated downregulation of MMP-2 activates the extrinsic apoptotic pathway in human glioma xenograft cells.. Int J Oncol.

[41] Cho SG, Choi EJ (2002). Apoptotic signaling pathways: caspases and stress-activated protein kinases.. J Biochem Mol Biol.

[42] Shih CM, Wu JS, Ko WC, Wang LF, Wei YH (2003). Mitochondria-mediated caspase-independent apoptosis induced by cadmium in normal human lung cells.. J Cell Biochem.

[43] Lee TJ, Kim EJ, Kim S, Jung EM, Park JW (2006). Caspase-dependent and caspase-independent apoptosis induced by evodiamine in human leukemic U937 cells.. Mol Cancer Ther.

[44] Cory S, Adams JM (2002). The Bcl2 family: regulators of the cellular life-or-death switch.. Nat Rev Cancer.

[45] Rao JS (2003). Molecular mechanisms of glioma invasiveness: the role of proteases.. Nat Rev Cancer.

[46] Kiyan J, Kiyan R, Haller H, Dumler I (2005). Urokinase-induced signaling in human vascular smooth muscle cells is mediated by PDGFR-beta.. EMBO J.

The article "Downregulation of uPAR and Cathepsin B Induces Apoptosis via Regulation of Bcl-2 and Bax and Inhibition of the PI3K/Akt Pathway in Gliomas" was retracted in 2020. Reasons: fabricated or falsified data; an official misconduct investigation; misconduct by an author; duplicated images.

[47] Duronio V (2008). The life of a cell: apoptosis regulation by the PI3K/PKB pathway.. Biochem J.

[48] Andrisani OM (1999). CREB-mediated transcriptional control.. Crit Rev Eukaryot Gene Expr.

[49] Pugazhenthi S, Nesterova A, Sable C, Heidenreich KA, Boxer LM (2000). Akt/protein kinase B up-regulates Bcl-2 expression through cAMP-response element-binding protein.. J Biol Chem.

[50] Finkbeiner S (2000). CREB couples neurotrophin signals to survival messages.. Neuron.

[51] Pugazhenthi S, Miller E, Sable C, Young P, Heidenreich KA (1999). Insulin-like growth factor-I induces bcl-2 promoter through the transcription factor cAMP-response element-binding protein.. J Biol Chem.

[52] Montminy MR, Bilezikjian LM (1987). Binding of a nuclear protein to the cyclic-AMP response element of the somatostatin gene.. Nature.

[53] Gondi CS, Lakka SS, Dinh D, Olivero W, Gujrati M (2004). Downregulation of uPA, uPAR and MMP-9 using small, interfering, hairpin RNA (siRNA) inhibits glioma cell invasion, angiogenesis and tumor growth.. Neuron Glia Biology.

[54] Gopinath S, Malla RR, Gondi CS, Alapati K, Fassett D (2010). Co-depletion of cathepsin B and uPAR induces G0/G1 arrest in glioma via FOXO3a mediated p27 upregulation.. PLoS One.

[55] Nalla AK, Gorantla B, Gondi CS, Lakka SS, Rao JS (2010). Targeting MMP-9, uPAR, and cathepsin B inhibits invasion, migration and activates apoptosis in prostate cancer cells.. Cancer Gene Ther.

[56] Brooks SA, Lomax-Browne HJ, Carter TM, Kinch CE, Hall DM (2010). Molecular interactions in cancer cell metastasis.. Acta Histochem.

[57] Mohamed MM, Sloane BF (2006). Cysteine cathepsins: multifunctional enzymes in cancer.. Nat Rev Cancer.

[58] Dasari VR, Veeravalli KK, Saving KL, Gujrati M, Klopfenstein JD (2008). Neuroprotection by cord blood stem cells against glutamate-induced apoptosis is mediated by Akt pathway.. Neurobiol Dis.

[59] Gopinath S, Vanamala SK, Gujrati M, Klopfenstein JD, Dinh DH (2009). Doxorubicin-mediated apoptosis in glioma cells requires NFAT3.. Cell Mol Life Sci.

[60] Wijsman JH, Jonker RR, Keijzer R, van d, V, Cornelisse CJ (1993). A new method to detect apoptosis in paraffin sections: in situ end-labeling of fragmented DNA.. J Histochem Cytochem.

[61] Gondi CS, Lakka SS, Dinh DH, Olivero WC, Gujrati M (2007). Intraperitoneal injection of an hpRNA-expressing plasmid targeting uPAR and uPA retards angiogenesis and inhibits intracranial tumor growth in nude mice.. Clin Cancer Res.

[62] Lakka SS, Gondi CS, Yanamandra N, Olivero WC, Dinh DH (2004). Inhibition of cathepsin B and MMP-9 gene expression in glioblastoma cell line via RNA interference reduces tumor cell invasion, tumor growth and angiogenesis.. Oncogene.

The article "Downregulation of uPAR and Cathepsin B Induces Apoptosis via Regulation of Bcl-2 and Bax and Inhibition of the PI3K/Akt Pathway in Gliomas" was retracted in 2020. Reasons: fabricated or falsified data; an official misconduct investigation; misconduct by an author; duplicated images.

[63] Gong J, Traganos F, Darzynkiewicz Z (1994). A selective procedure for DNA extraction from apoptotic cells applicable for gel electrophoresis and flow cytometry.. Anal Biochem.

